The article "Study on Nursing Effect of Psychological Intervention on Uremic Hemodialysis Patients" was retracted in 2023. Reasons: unreliable results or conclusions; lack of ethics approval or compliance; concerns about the data; concerns about the peer review.

# Study on Nursing Effect of Psychological Intervention on Uremic Hemodialysis Patients

**DOI:** 10.1155/2022/8040656

**Published:** 2022-07-13

**Authors:** Yan Chen, Jie Ding, Chunqing Li, Ting Wu, Qingya Li, Rujing Chen, Jingfen Zhou

**Affiliations:** ^1^Nephrology Department, The Affiliated Hospital of Jiangnan University, 214000, China; ^2^Hematology Department, The Affiliated Hospital of Jiangnan University, 214000, China

## Abstract

**Aim:**

Patients in the hemodialysis stage are prone to psychological pressure of depression and anxiety and have resistance, which affects the clinical treatment effect. Effective psychological intervention plays a very important role in improving patients' psychological pressure and patients' compliance. The aim of this study is to explore the nursing effect of psychological intervention on uremic hemodialysis patients.

**Methods:**

There were 126 uremic hemodialysis patients admitted to the hospital from August 2020 to December 2021. The patients were randomly divided into the routine nursing care group (*n* = 63) and psychological intervention group (*n* = 63). The routine nursing care group received routine nursing care for uremia hemodialysis patients. The psychological intervention group implemented psychological intervention on uremia hemodialysis patients. The methods of psychological intervention mainly include establishing a good nurse-patient relationship, popularizing hemodialysis knowledge, timely psychological counseling for patients, and organizing patient communication meetings. The treatment compliance, Self-rating Anxiety Scale (SAS) and Self-rating Depression Scale (SDS) of the two groups were compared before and after nursing. SF-36 scale was used to evaluate the quality of life of patients. The incidence of complications and nursing satisfaction were compared between the two groups.

**Results:**

The treatment compliance rate and nursing satisfaction of hemodialysis uremic patients in the psychological intervention group were significantly higher than the routine nursing care group. The SAS and SDS of hemodialysis uremia patients in the psychological intervention group were significantly lower than the routine nursing care group after psychological intervention, and SF-36 scale was significantly higher than the routine nursing group. The main complications of uremic hemodialysis patients are hypotension, hyperkalemia, internal fistula occlusion, and infection. Compared with the routine nursing care group, the incidence of complications in the psychological intervention group was significantly reduced.

**Conclusion:**

The implementation of psychological nursing intervention for uremic hemodialysis patients have a very significant effect on reducing the incidence of complications and improving anxiety, depression, treatment compliance, and the quality of life and the nursing satisfaction.

The article "Study on Nursing Effect of Psychological Intervention on Uremic Hemodialysis Patients" was retracted in 2023. Reasons: unreliable results or conclusions; lack of ethics approval or compliance; concerns about the data; concerns about the peer review.

## 1. Introduction

Uremic patients are in the end stage of renal failure. Hemodialysis is mainly used for alternative treatment to replace the excretory function of the kidney, ensure the normal metabolism of the body, and prolong the survival time of patients [1–3].

Hemodialysis treatment is a relatively long-term process. During hemodialysis, patients not only need to bear a large economic burden but also the possible complications during renal dialysis [4, 5]. Patients are prone to psychological pressure of depression and anxiety and resist hemodialysis, which affect the clinical treatment effect. If we cannot get timely and effective counseling and nursing intervention, the continuous bad psychological state is easy to develop into anxiety disorder and depression, which will have a negative impact on the quality of life of patients. Studies have shown that the incidence of depressive symptoms in uremic patients is 68.8%, which is basically the same as 68.0% found abroad, slightly higher than 55.5% found by domestic researchers, and the incidence of anxiety symptoms is 67.25%, higher than 51.0% found abroad [6–8]. Therefore, psychological intervention for uremic hemodialysis patients is of great significance to the therapeutic effect of patients.

Psychological intervention refers to the planned and purposeful implementation of psychological counseling for the intervention object with the help of professional psychological counseling personnel, so as to reduce psychological pressure and complete the predetermined goal [9, 10]. Effective psychological intervention plays a very important role in improving patients' psychological pressure and improving patients' compliance [11–13]. This study collected uremic hemodialysis patients and implemented psychological intervention to explore the nursing efficacy of psychological intervention on uremic hemodialysis.

## 2. Materials and Methods

### 2.1. Patients

There were 126 uremic hemodialysis patients admitted to the hospital from August 2020 to December 2021. According to the random number table method, the patients were randomly divided into the routine nursing group (*n* = 63) and psychological intervention group (*n* = 63). The routine nursing care group received routine nursing care for uremia hemodialysis patients. The psychological intervention group implemented psychological intervention on uremia hemodialysis patients.

### 2.2. Inclusion Criteria

The patients were diagnosed with uremia and required hemodialysis. The patients had no medical history or previous medical history. The patient is conscious and communicable. The patients and their families gave informed consent and signed the informed consent form voluntarily.

The article "Study on Nursing Effect of Psychological Intervention on Uremic Hemodialysis Patients" was retracted in 2023. Reasons: unreliable results or conclusions; lack of ethics approval or compliance; concerns about the data; concerns about the peer review.

### 2.3. Exclusion Criteria

Patients had severe functional diseases of other organs or mental disorders. Patients withdrew from the study.

### 2.4. Nursing Methods

The routine nursing care group patients were treated with routine nursing methods. The psychological intervention group patients were implemented psychological intervention on the basis of the routine nursing care group. The methods of psychological intervention mainly include the ways of psychological intervention, mainly including establishing a good nurse-patient relationship, popularizing hemodialysis knowledge, timely psychological counseling for patients, and organizing patient communication meetings. Nurses need to fully understand the specific situation of patients, including the course of disease, condition, personality characteristics of patients, economic and living conditions, and family background. On this basis, winning the trust of patients and their families through conversation and other skills, popularizing patients' disease knowledge, explain in detail the harm of negative emotions to the disease, and pushing pictures and videos among patients, so as to provide convenience for patients to learn. For example, establishing a WeChat patients group, timely publish health information in the group, and improve patients' treatment compliance. They listen to the patient's negative psychological experience sincerely and patiently. Patients had a process from denying the disease to negative reaction. According to this characteristic, we should guide patients to gradually accept their condition and actively respond to psychological nursing interventions. The main method is the acceptance-based therapy in cognitive behavioral therapy, which focuses on letting patients change the negative psychology of “my life is over,” gradually accept their condition, actively cooperate with the treatment, and rekindle the hope of life. We regularly organize patients to participate in “communication meetings,” simulate the impact of negative emotions on patients through scenario simulation, discuss how to solve problems, and encourage patients to actively face diseases and optimistic treatment.

### 2.5. Observation Index

To investigate the treatment compliance rate and nursing satisfaction of patients in the routine nursing care group and the psychological intervention group. Treatment compliance can be divided into complete compliance, partial compliance, and noncompliance. Complete compliance means that the patient can fully follow the doctor's advice. Partial compliance refers to the patient's partial implementation of the doctor's order. Noncompliance refers to failure to cooperate with treatment. The treatment compliance rate is the sum of the proportion of complete compliance and partial compliance. The nursing satisfaction of patients was investigated. The evaluation results included very satisfied, satisfied, basically satisfied, and dissatisfied. The anxiety and depression of patients in the routine nursing care group and the psychological intervention group before and after nursing were counted. The patient's anxiety was assessed by Self-rating Anxiety Scale (SAS). The patient's depression was assessed by Self-rating Depression Scale (SDS). The SAS includes 20 items, with a total score of 100. The higher the SAS, the more serious of the anxiety. The SDS includes 20 items, with a total score of 100. The higher the SDS, the more serious of depression. The complications were observed of the two groups. SF-36 was used to evaluate the quality of life of patients before and after intervention. SF-36 includes physiological function, mental health, vitality, emotional function, social function, and physical pain. The total score is 100. The higher the score, the better the quality of life.

The article "Study on Nursing Effect of Psychological Intervention on Uremic Hemodialysis Patients" was retracted in 2023. Reasons: unreliable results or conclusions; lack of ethics approval or compliance; concerns about the data; concerns about the peer review.

### 2.6. Statistical Analysis

The data were statistically analyzed using SPSS 23.0. Measurement data were presented as mean ± variance. Two groups were compared using *t*-test. Count data were presented in cases (%). The chi-square test was used to compare the two groups. *P* < 0.05 means the difference is statistically significant.

## 3. Results

### 3.1. Basic Clinical Characteristics of Patients

In the routine nursing care group, there were 34 male patients and 29 female with an average age of 57.32 ± 8.64 years, ranging from 42 to 75 years old. The average time of hemodialysis was 1.04 ± 0.11 years, ranging from 0.25 to 1.5 years. There were 36 males and 27 females in the psychological intervention group, with an average age of 57.32 ± 8.64 years, ranging from 41 to 73 years old. The average time of hemodialysis was 1.06 ± 0.10 years, ranging from 0.3 to 1.5 years. There was no significant difference in equal general data between the two groups, but the comparability was strong (*P* > 0.05).

### 3.2. The Treatment Compliance of Patients

The results showed that the treatment compliance rate of hemodialysis uremic patients in the psychological intervention group was significantly higher than the routine nursing care group (Table 1). This showed that the implementation of psychological intervention nursing can effectively improve the treatment compliance of hemodialysis patients.

The article "Study on Nursing Effect of Psychological Intervention on Uremic Hemodialysis Patients" was retracted in 2023. Reasons: unreliable results or conclusions; lack of ethics approval or compliance; concerns about the data; concerns about the peer review.

### 3.3. Incidence of Postoperative Complications in Patients

The main complications of uremic patients in hemodialysis included hypotension, hyperkalemia, internal fistula occlusion, and infection. The incidence of complications in the psychological intervention group was significantly lower than the routine nursing care group (Table 2).

### 3.4. Comparison of SAS and SDS of Patients

The SAS (Figure 1(a)) and SDS (Figure 1(b)) of uremic hemodialysis patients were compared between the psychological intervention group and the routine nursing care group before and after nursing. Before nursing, there were no significant difference in SAS and SDS between the routine nursing care group and the psychological intervention group. After receiving nursing care, the SAS and SDS of uremic hemodialysis patients in the two groups decreased. Compared with the uremic hemodialysis patients in the routine nursing care group, the SAS and SDS of uremic hemodialysis patients in the psychological intervention group were significantly lower. This showed that psychological intervention can significantly alleviate the anxiety and depression of uremic hemodialysis patients.

### 3.5. Comparison of Patients' Quality of Life

The quality of life of uremic hemodialysis patients was compared between the psychological intervention group and the routine nursing care group. After receiving nursing care, the quality of life of uremic hemodialysis patients in the two groups showed different degrees of improvement, and the scores of uremic hemodialysis patients in the psychological intervention group were significantly better than that in the routine nursing care group (Figure 2).

### 3.6. Nursing Satisfaction of Patients

The nursing satisfaction of uremic hemodialysis patients was compared between the psychological intervention group and the routine nursing care group. Compared with the uremic hemodialysis patients in the routine nursing care group, the nursing satisfaction of uremic hemodialysis patients in the psychological intervention group was significantly higher (Table 3). The above results showed that the implementation of psychological intervention has a significant effect on improving the nursing satisfaction of uremic hemodialysis patients.

## 4. Discussion

Uremia is a series of poisoning symptoms when acute or chronic renal insufficiency develops to a serious stage, often accompanied by water, electrolyte disorder, endocrine dysfunction, and other symptoms, which poses a serious threat to the life safety of patients [14–16]. Hemodialysis is one of the important treatment methods for patients with uremia, which can effectively improve the survival rate of patients. It is affected by economic conditions and physical aspects. Moreover, most patients do not know enough about treatment knowledge, resulting in negative emotions [17–19]. Relevant studies have shown that the common problems in hemodialysis patients are anxiety and depression, which seriously affect the treatment of patients [20, 21]. How to reduce patients' negative emotions through effective nursing has become a key topic of clinical medical staff.

The article "Study on Nursing Effect of Psychological Intervention on Uremic Hemodialysis Patients" was retracted in 2023. Reasons: unreliable results or conclusions; lack of ethics approval or compliance; concerns about the data; concerns about the peer review.

The traditional nursing intervention is mainly aimed at the basic nursing method adopted in the process of disease treatment, which is difficult to effectively eliminate the psychological pressure and negative emotions of patients [22–24]. Psychological nursing intervention focuses on taking targeted intervention measures according to the psychological state of patients. First of all, we need to accurately evaluate the psychological state of patients, formulate scientific and reasonable psychological intervention plans and measures according to the evaluation results, and carry out effective psychological counseling through communication [25–27]. Popularizing patients' disease knowledge, explaining in detail the harm of negative emotions to the disease, and pushing pictures and videos among patients provide convenience for patients to learn. At the same time, we regularly organize patients to participate in “communication meetings,” simulating the impact of negative emotions on patients through scenario simulation, discussing how to solve problems, and encouraging patients to actively face the disease and treat optimistically [28–30]. By taking various intervention measures to relieve the anxiety and tension of patients, improve treatment compliance, and effectively improve the treatment effect [31–33], the results of this study showed that the treatment compliance of patients receiving psychological intervention was significantly increased, and the incidence of complications was significantly reduced.

This study found that through psychological nursing intervention, the degree of depression and anxiety of uremic patients was significantly reduced and the quality of life was significantly improved. Depression is characterized by depression, accompanied by negative beliefs and pessimism. Anxiety reflects the patient's concern about the future development direction of the disease. For uremic patients, they often have a sense of helplessness, that is, they are unwilling to accept the fact of illness. This idea makes patients fall into a negative dilemma [34–36]. In addition, the long-term nature of uremic treatment and the burden of treatment costs will also aggravate patients' loss of confidence in treatment [37, 38]. Therefore, the key to psychological care for patients with uremia is to let patients accept it slowly from unwilling to accept it, change their negative cognition of their life, and let patients understand that uremia can live like healthy people through treatment, so as to stimulate patients' confidence in active treatment and good life [39–41]. The method adopted in this study is a new branch of cognitive behavioral therapy, that is, reception-based therapy, which is aimed at helping the treatment object accept and actively deal with their own psychological problems [42, 43]. Acceptance-based cognitive behavioral therapy can effectively alleviate the anxiety and depression of uremic hemodialysis patients. In addition, the communication frequency between similar patients should be increased in addition to the psychological intervention directly carried out by nurses. The mutual conversation and encouragement of the mutual aid group will further strengthen the patients' awareness of active treatment.

The article "Study on Nursing Effect of Psychological Intervention on Uremic Hemodialysis Patients" was retracted in 2023. Reasons: unreliable results or conclusions; lack of ethics approval or compliance; concerns about the data; concerns about the peer review.

In conclusion, the implementation of psychological intervention for uremic hemodialysis patients can help patients improve their cognition of active treatment, treatment compliance, the degree of anxiety and depression, and the nursing satisfaction. Therefore, it is worth popularizing on clinic. For the wide application of psychological intervention methods in clinic, we still need to further carry out multicenter and large-sample research and further improve the scheme of psychological intervention.

## Figures and Tables

**Figure 1:** Comparison of SAS (a) and SDS (b) of uremic hemodialysis patients in the psychological intervention group and the routine nursing care group before and after nursing. ^∗^*P* < 0.05.

**Figure 2:** Comparison of SF-36 scale scores between the psychological intervention group and the routine nursing care group during uremia hemodialysis. ^∗^*P* < 0.05.

**Table 1:** Comparison of treatment compliance rate of the uremic hemodialysis patients between the routine nursing care group and the psychological intervention group (*n* (%)).

Group	*n*	Complete compliance	Partial compliance	Noncompliance	Compliance rate
Psychological intervention group	63	42 (66.67)	18 (28.57)	3 (4.76)	60 (95.24)
Routine nursing care group	63	34 (53.97)	16 (25.40)	13 (20.63)	50 (79.37)
*X* ^2^		7.210			
*P*		0.027			

**Table 2:** Comparison of complications between the two groups (*n* (%)).

Group	*n*	Hypotension	Hyperkalemia	Internal fistula occlusion	Infection
Psychological intervention group	63	1 (1.59)	1 (1.59)	2 (3.17)	2 (3.17)
Routine nursing care group	63	4 (6.35)	3 (4.76)	3 (4.76)	5 (7.94)
*X* ^2^		4.629			
*P*		0.031			

The article "Study on Nursing Effect of Psychological Intervention on Uremic Hemodialysis Patients" was retracted in 2023. Reasons: unreliable results or conclusions; lack of ethics approval or compliance; concerns about the data; concerns about the peer review.

**Table 3:** Comparison of nursing satisfaction between the uremic hemodialysis patients in the routine nursing care group and the psychological intervention group (*n* (%)).

Group	*n*	Very satisfied	Satisfied	Basically satisfied	Dissatisfied	Degree of satisfaction
Psychological intervention group	63	35 (55.56)	17 (26.98)	7 (11.11)	4 (6.35)	59 (93.65)
Routine nursing care group	63	26 (41.27)	11 (17.46)	14 (22.22)	12 (19.05)	51 (80.95)
*X* ^2^		8.947				
*P*		0.030				

## Data Availability

No data were used to support this study.
